# GREB1 Functions as a Growth Promoter and Is Modulated by IL6/STAT3 in Breast Cancer

**DOI:** 10.1371/journal.pone.0046410

**Published:** 2012-10-03

**Authors:** Mingli Liu, Guangdi Wang, Carmen R. Gomez-Fernandez, Shanchun Guo

**Affiliations:** 1 Department of Microbiology, Biochemistry and Immunology, Morehouse School of Medicine, Atlanta, Georgia, United States of America; 2 Department of Chemistry, Xavier University of Louisiana, New Orleans, Louisiana, United States of America; 3 Department of Pathology, Department of Medicine, University of Miami School of Medicine, Miami, Florida, United States of America; Virginia Commonwealth University, United States of America

## Abstract

**Background:**

**G**rowth **R**egulation by **E**strogen in **B**reast cancer (GREB1) was an estrogen receptor (ER) target gene, and GREB1 expression inversely correlated with HER2 status, possibly as a surrogate marker for ER status and a predictor for tamoxifen resistance in breast cancer patients. In the present study, we examine the function and regulation of GREB1 in breast cancer, with the goal to develop GREB1 as a biomarker in breast cancer with de novo and acquired tamoxifen resistance.

**Methods:**

We overexpressed GREB1 using adenovirus containing the full length GREB1 cDNA (Ad-GREB1) in breast cancer cell lines. The soft agar assay was used as a measure of anchorage independent growth. The effects of GREB1 on cell proliferation in MCF-7 cells transduced with Ad-GREB1 were also measured by the me olic activity using AlamarBlue assay. We tested whether there was interaction between STAT3 and ER, which could repress GREB1 expression by immunoprecipitation assay. The effects of IL-6/JAK/STAT3 cascade activation on estrogen-induced GREB1 promoter activity were determined by luciferase assay and those on gene expression were measured by real time reverse transcription polymerase chain reaction (qRT-PCR).

**Results:**

We found that the ability of breast cancer cells to grow in soft agar is enhanced following GREB1 transfection. In MCF-7 cells transduced with Ad-GREB1 or transfected with siRNA GREB1, the metabolic activity was increased or completely abolished, suggesting that GREB1 may function as a growth promoter in breast cancer. E2 treatment increased GREB1 promoter luciferase activity. IL-6 inhibited E2-induced GREB1 transcription activity and GREB1 mRNA expression. Constitutively expressing active STAT3 construct (STAT3-C) dramatically decreased GREB1 transcription.

**Conclusions:**

These data indicate that overexpression of GREB1 promotes cell proliferation and increases the clonogenic ability in breast cancer cells. Moreover, Il6/STAT3 modulates estrogen-induced GREB1 transcriptional activity in breast cancer cells.

## Introduction

Current endocrine therapies for breast cancer patients target the estrogen receptor (ER) by reducing its ligand-induced activation, blocking its function and ultimately inducing ER degradation. Although these therapies are effective in many patients with ER-positive tumors, long-term follow up and clinical trials have demonstrated that up to 62% of breast cancers that are initially responsive to endocrine therapy eventually relapse, with the patients then requiring salvage surgery [1], [2], [3]. Therefore, identification of molecular markers that can predict responses to anti-estrogen therapy in ER positive breast cancer is critically needed.

Tamoxifen treatment is the most frequently utilized therapy for patients with estrogen receptor α (ERα) positive breast cancer. Although many patients benefit from tamoxifen, one-third of ERα positive (ER+) breast cancers exhibit primary resistance to tamoxifen treatment (intrinsic, or de novo resistance) [4]. The remaining 70% of ER-positive breast cancers initially respond to the tamoxifen but have a great tendency to relapse and subsequently fail to respond to tamoxifen (acquired resistance) [5], [6]. Tamoxifen competes with estrogen for ER binding sites and functions as an antagonist of ER [6]. Binding of tamoxifen to ERα results in conformational changes of the receptor, thereby impairing the ability of ERα to recruit coactivators or corepressors to the tamoxifen-ER complex [6]. The interaction between tamoxifen and ER not only determines the antagonist effects of tamoxifen on the tissues, but also indicates possible mechanisms by which resistance might develop in breast cancer. A better understanding of the biological and molecular mechanisms underlying intrinsic and acquired tamoxifen resistance could provide novel strategies to circumvent resistance to tamoxifen, and aid in the optimal design of order and duration of endocrine reagents for further improvements in disease outcomes.

Numerous predictive and prognostic factors for endocrine response have been evaluated in breast cancer. Established biomarkers such as ER and progesterone receptor (PgR) are important positive predictive markers for response to endocrine therapy in patients with breast cancer [7]. Total loss of PgR predicts relative resistance to the anti-estrogen tamoxifen, but may not indicate resistance to aromatase inhibitors [8]. New adjuvant setting studies also indicate that high levels of epidermal growth factor receptor 2 (HER2) is associated with tamoxifen resistance, but not resistance to aromatase inhibitors [8]. Ki67, a typical although modest prognostic factor, has recently been recognized as a more effective predictor of treatment efficacy for both endocrine and chemotherapy [9]. An estrogen targeted gene Zinc transporter LIV-1 (SLC39A6) was recently shown to be associated with Ki67 conferring resistance to tamoxifen and fulvestrant [9]. New clinical studies indicate NF-κB p50 activation as a potential prognostic marker capable of identifying a high-risk subset of primary ER-positive breast cancer destined for early relapse in spite of adjuvant tamoxifen therapy. The sensitivity to tamoxifen can be restored by interrupting activation of NF-κB [10], [11]. ErbB3 has also played an important role in the development of resistance to antiestrogens such as tamoxifen [12]. Since the inception and broad application of DNA microarray technology, numerous multigene expression profiling assays have been developed with the aim of identifying new prognostic biomarkers predicting response to endocrine therapy. Among them, the Oncotype DX assay and the MammaPrint profile are currently undergoing clinical evaluation to determine their efficacy [7]. Gene expression signatures suggest that a “proliferation cluster” including Ki-67, proliferating cell nuclear antigen (PCNA), some proliferation-related genes and cell cycle genes may be the strongest predictor for metastasis and relapse in tamoxifen treated ER-positive breast cancer patients, emphasizing the important roles of proliferation genes in prognosis [13], [14], [15]. Although biomarkers as described above appear to be of certain biological importance, only few such as ER, PgR and HER2 have proven clinically applicable. We have reported that GREB1 correlates with ERα expression in breast cancer cell lines and breast cancer tissues [16]. However, in several anti-estrogen resistant cell lines including BT-474, T47D and SUM44, which are ER-positive, GREB1 expression is either reduced or absent. It has been well documented that there is interplay between HER2 activity and loss of ER transcription [17], and anti-estrogen resistant tumors are characterized by elevated HER2 levels [18], [19], [20]. Consistent with these findings, we have reported that GREB1 expression inversely correlated with HER2 expression in ER-positive breast cancer patients. In other words, ER-positive, GREB1-negative patients have a significantly greater tendency to positively express HER2 protein compared to ER-positive, GREB1-positive patients [21]. Patients with GREB1 positive expression exhibit significant tamoxifen sensitivity and prolonged survival compared to the patients with GREB1 negative expression [22]. In addition, we also showed previously that not only GREB1 but also other ER-regulated genes such as IGFBP4, IRS-1 and BCL-2 mRNA expressions were increased as HER2 signaling was blocked, suggesting that HER2 may regulate GREB1 through ER pathways [21]. However very little is known about the function of GREB1 and the mechanism by which it is regulated by ER. Earlier reports indicated that signal transducer and activator of transcription (STAT3) acts downstream of HER2 [23], [24]. STAT3 is tyrosine phosphorylated through the interleukin-6 (IL-6)/glycoprotein 130/Janus kinase pathway in breast cancer [25]. STATs and ER can physically interact in vivo [26], [27]. In the present study, we investigated the function of GREB1 gene on cell proliferation and trasnfrormation and whether the HER2 downstream signaling molecule STAT3 regulates ER transcription resulting in negative or decreased expression of GREB1 in breast cancer cells. We believe that our study will provide a basis for development of GREB1 as a novel biomarker in combination with ER to better identify breast cancer patients who will benefit from tamoxifen therapy and those who will likely develop resistance to endocrine therapy.

## Results

### GREB1 is Induced by E2 in ER-positive Breast Cancer Cell Line

GREB1 was detected in MCF-7 cells treated with E2 for 24 and 48 hrs, while no protein is detected in the ER-negative BT-549 cells or in MCF-7 cells grown in estrogen-free conditions in Western blotting assay (Figure 1A). Treatment with ICI 182,780 (ICI), an estrogen receptor antagonist, and silencing the GREB1 gene by siRNA led to the loss of GREB1 protein expression. As shown in Figure 1B, GREB1 protein expression is reduced in MCF-7 cells treated with estrogen plus ICI 182,780 compared to that observed in cells treated with estrogen alone. Figure 1C shows the loss of detectable GREB1 protein when GREB1 is knocked down by GREB1 siRNA (SiGREB1) at 48 hours compared to control (CSiRNA), CSiRNA has no effect on E2-induced GREB1 production. Corresponding densitometric analysis of the bands performed with the ImageQuant program (Bio-Rad) areshown below the Western blot. E2-induced GREB1mRNA levels were similarly analyzed as above, with GREB1 mRNA levels correlating well with GREB1 protein expressions. Upon E2 stimulation, GREB1 mRNA is notable as early as 24 hours and lasts up to 48 hours as presented in a time course study in Figure 1D. BT-549 cells express GREB1 mRNA as low as the control. ICI treatment (Figure 1E) and silencing the GREB1 gene (Figure 1F) both significantly reduced the GREB1 expression at the transcriptional level.

**Figure 1:** GREB1 is induced by E2 in ER-positive breast cancer cell lines. A, Western blotting detects a single band of ∼216 kD in E2-deprived MCF-7 cells treated with estrogen for 24 and 48 hrs while no protein is detected in the ER-negative BT-549 cells or in MCF-7 cells grown in estrogen-free conditions. B, GREB1 protein expression was reduced in the MCF-7 cells treated with estrogen plus ICI 182,780 (ICI) compared to that observed in cells treated with estrogen alone. C, Figure C shows loss of detectable GREB1 protein when GREB1 is knocked down by GREB1 siRNA (SiGREB1) at 48 hours. Control siRNA (CSiRNA) has no effect on E2-induced GREB1 production. Corresponding densitometric analysis of the bands performed with the ImageQuant program (Bio-Rad) were shown below the Western blot. E2-induced GREB1mRNA levels were also analyzed, GREB1 mRNA levels were well correlated with GREB1 protein expressions. D, GREB1 mRNA is notable as early as 24 hours and lasts up to 48 hours as presented in a time course study. BT-549 cells express GREB1 mRNA as low as the control. E and F, ICI treatment (Figure 1E) and silencing the GREB1 gene (Figure 1F) significantly reduced the GREB1 expression at transcriptional level. Data are shown as mean ± SD. *P<0.05; **P<0.01.

### GREB1 mRNA Correlates with ER Status in Breast Cancer Patients, and Predicts Patient Survival and Responses to Tamoxifen Treatment

GREB1 is the most sensitive ER-regulated gene in response to E2 stimulation in breast cancer patients [28]. ERα is the prototypic phenotypic marker used in prognosis of breast cancer and it directly controls GREB1 expression [29], [30]. Furthermore, GREB1 is tightly correlated with ERα expression in breast cancer cell lines and it is required for breast cancer cell growth [28], [31]. However, GREB1 as a cancer biomarker and the clinical significance of GREB1 protein expression in human breast cancer is underexplored. GREB1 function and regulation need to be fully investigated. To this end, we analyzed GREB1 expression in publicly available breast cancer microarray studies using the Oncomine database and gene microarray data analysis tool [32], [33]. Meta-analysis of microarray gene expression data sets related to human cancer genes revealed that GREB1 mRNA is highly expressed in breast carcinomas compared to normal breast tissues (T-test: 4.815; P-value: 2.1E-5) (Figure 2A) [34]. Using the same Oncomine research platform, microarray data obtained from 2321 patients of human breast cancer patients (1651 ER-positive, 670 ER-negative) through 15 studies were also evaluated for the relationship between GREB1 expressions and other clinical parameters. Meta-analysis from published database demonstrated that GREB1 expression is significantly increased in ER-positive cancer patients compared to ER-negative cancer patients (Figure 2B) [34], [35], [36], [37], [38], [39], [40], [41], [42], [43], [44], [45], [46], [47]. We further analyzed the effects of GREB1 mRNA on patients’ survival using the data from the North Central Cancer Treatment Group Trial, Tamoxifen (TAM) arm of 89-30-52 which recruited 225 patients (Phase III trial of adjuvant therapy with Tamoxifen alone or combined with Fluoxymesterone in postmenopausal women with resected estrogen receptor positive breast cancer) [48], [49], [50]. Although PgR expression alone has historical precedence as a clinical prognosticator of breast cancer patient in response to hormone therapy [8], [51], [52], the analysis showed that GREB1 mRNA predicts disease-free survival (DFS) in Tamoxifen-treated patients better than PgR or ER (Table 1). This assessment of clinical relevance was further corroborated in a patient survival analysis using an online database containing the expression of 22,277 genes and 20-year survival information of 1809 patients [53]. The database has recently been updated to include survival information of 2898 breast cancer patients (http://www.kmplot.com/analysis/). GREB1 downregulation was found to correlate strongly with poor relapse free survival (RFS) for all breast cancer patients followed for 20 years (Fig. 2C, hazardous ratio 0.66, *p* = 1.1×10^−10^). For patients with ER+ breast tumor, lower expression of GREB1 was also seen as significantly associated with decreased survival (Fig. 2D, hazardous ratio 0.75, *p* = 0.0029). As shown in Fig. 2E, for ER+ patients who have received endocrine therapy, reduced GREB1 expression predicts worse outcome in RFS (hazardous ratio 0.63, *p* = 0.041).

**Table 1:** 225 patients from the TAM arm of 89-30-52.

		Log-rank Test Results, when factor dichotomized at its median value		
	Median (range)	OS (n = 87 events)	DFS (n = 97 events)	TTBR (n = 43 events)
GREB1	−3.00 (−9.99 to −0.14)	P = 0.038	P = 0.023	P = 0.038
ER	0 (−8.59 to 2.31)	P = 0.365	P = 0.434	P = 0.646
PR	−4.21 (−10.85 to 0.81)	P = 0.108	P = 0.140	P = 0.056

OS- death due to any cause.

Disease-free survival (DFS). Disease-free survival was defined as the time from randomization to the documentation of the first adverse event where an adverse event is defined as local, region, or distant disease progression, the development of contralateral breast disease, or death from any cause without documentation of another adverse event.

Time to breast cancer recurrence (TTBR). Time to breast cancer recurrence was defined as the time from randomization to the documentation of the first adverse breast event where an adverse breast event is defined as local, region, or distant disease progression.

**Figure 2:** GREB1 mRNA correlates with ER status in breast cancer patients, and predicts responses in Tamoxifen-treated patients. Meta-analysis was performed using the Oncomine Research Platform- based microarray studies. A. Microarray analysis of 7 normal breast tissues (red bar) and 40 breast cancers (blue bar). The mean values of GREB1 mRNA expression are shown here. B. Microarray analysis of 2321 patients (1651 ER-positive, 670 ER-negative). The level of GREB1 expression is higher in ER-positive breast cancer patients, which are depicted by red-colored bars and ER-negative patients are represented by blue ones. Kaplan-Meier survival plots demonstrate the prognostic relevance of GREB1 expression on patient survival using various data cohorts. C. Reduced expression of GREB1 is predictive of lower relapse free survival (HR = 0.66, *p* = 1.1×10^−10^) for all patients; D. For ER+ breast cancer patients, lower GREB1 expression is correlated with decreased relapse free survival (HR = 0.75, *p* = 0.0029); E. Endocrine treated ER+ breast cancer patients have reduced relapse free survival if their tumors expressed lower GREB1 level (HR = 0.63, *p* = 0.041).

### GREB1 is Localized in the Nucleus in ER-positive Breast Cancer Cell Line and Breast Cancer Tissues

The immunofluorescence staining was performed to determine the subcellular localization of GREB1 protein. E2-deprived MCF-7 cells were treated with 1 nM E2 for 24 h and then stained for GREB1 in red (Alexa Fluor® 555, Figure 3A) and nucleus in blue (DAPI, Figure 3B). The merged picture is given in Figure 3C, which demonstrates a clear nuclear localization of GREB1 (there are some specks of GREB1 proteins in the surrounding cytoplasm, but GREB1 appears mostly nuclear). Figure 3D to 3F show staining of negative control lacking primary antibody GREB1. The nuclear localization of GREB1 was further confirmed by introducing exogenous GREB1 into MCF-7 cells. We overexpressed GREB1 using adenovirus containing the full length GREB1 cDNA in estrogen-deprived MCF-7 breast cancer cells. E2-deprived MCF-7 cells were infected with Ad-CMV-null and Ad-GREB1 at a MOI of 10. After 72 h, the cells were stained for GREB1 in red (Alexa Fluor® 555, Figure 3G) or nucleus in blue (DAPI, Figure 3H), the merged image is shown in Figure 3I. Figure 3J to 3L show the staining of Ad-CMV-null as negative control. There was low background in the negative controls, however MCF-7 cells showed a significant efficiency of nuclear transfection of Ad-GREB1 compared with the transfection of empty vector (Fig. 3J to 3L). Immunohistochemistry staining (IHC) of ER-positive MCF-7 cells (Figure 3M, 3N) and ER-positive breast cancer tissues (Figure 3Q) confirmed the observation of GREB1 nuclear localization obtained from immunofluorescent staining described as above. ER-negative breast cancer cell line MDA-MB-231 and ER-negative breast cancer tissues expressed undetectable levels of GREB1 (Figure 3O, P and R). Therefore, both immunofluorescence and IHC staining results show that GREB1 is localized predominantly to the nucleus in both ER-positive breast cancer cell line and ER-postive primary breast cancer tissues.

**Figure 3:** GREB1 is localized in the nucleus in ER-positive breast cancer cell line and breast cancer tissues. Subcellular localization of GREB1 in breast cancer cells was determined by immunofluorescent microscopy and immunohistochemical staining (IHC). A to C, E2-deprived MCF-7 cells were stimulated with E2 for 24 h and then stained for GREB1 in red (Alexa Fluor 555, A) and nucleus in blue (DAPI, B), and C gave the merged picture. GREB1 is almost exclusively localized in the nucleus. D to F showed staining of negative control lacking primary GREB1 antibody. The nuclear localization of GREB1 was further confirmed by introducing exogenous GREB1 into MCF-7 cells. GREB1 was stained in red in Figure 3G, nucleus was stained in blue in Figure 3H, the merged image was shown as Figure 3I. Figure 3J to 3L showed the staining of negative control. IHC staining showed that ER-positive MCF-7 cells (Figure 3M) and ER-positive breast cancer tissues (Figure 3Q) detected GREB1 expression (brown). ER-negative breast cancer cell line MDA-MB-231 (Figure 3O) and ER-negative breast cancer tissues expressed undetectable levels of GREB1 (Figure 3R). HE staining was also showed for ER-positive breast cancer (Figure 3N) and ER-negative breast cancer (Figure 3P).

### Overexpression of GREB1 Promotes Cell Proliferation and Increases the Clonogenic Ability of Breast Cancer Cells

To investigate the biological functions of GREB1 in tumor formation and progression, we tested the effects of overexpression of GREB1 on breast cancer cell growth. We overexpressed GREB1 using adenovirus vector containing the full length GREB1 cDNA, which has been shown to significantly improve transfection efficiency. We checked the transfection efficiency using quantitative reverse transcription polymerase chain reaction (qPCR) analysis. Briefly, MDA-MB-231, MDA-MB-453, MDA-MB-468 and 3-day estrogen depleted MCF-7 were infected with Ad-CMV-null and Ad-GREB1 at an MOI of 10, respectively. After 24 h, the cells were lysed and the expression of GREB1 mRNA in infected cells was analyzed by qPCR assay. Our results showed that the cells transduced with Ad-GREB1 express high GREB1 mRNA levels, whereas GREB1 was at non detectable level in all cells including estrogen deprived MCF-7 asynchronous cultures (Figure 4D, middle upper panel), MDA-MB-231 (Figure 4A, right upper panel), MDA-MB-453 (Figure 4B, right upper panel), and MDA-MB-468 (Figure 4C, right upper panel) cell cultures transduced with empty vector. Subsequently, the soft agar assay was used as a measure of anchorage independent growth, a defining characteristic of transformed cells. We found that the ability of MDA-MB-231 (Figure 4A, left panel), MDA-MB-453 (Figure 4B, left panel), MDA-MB-468 (Figure 4C, left panel), and MCF-7 (Figure 4D, middle lower panel) to grow in soft agar is substantially enhanced by 1.9-, 2.2-, 1.7- and 2.0- fold following GREB1 transfection. We next tested E2 deprived MCF-7 cells for the effects of GREB1 on cell proliferation. In parallel, cells were also treated with vehicle and estradiol (E2) as controls. On day 4, the mitogenic effects were measured using an AlamarBlue reduction assay. The growth rate in MCF-7 cells treated with E2 is 3.5 fold higher than in estrogen depleted, quiescent controls. Transfection with the SiGREB1 had marked effect on cells treated with E2, as cell proliferation was completely abolished (Figure 4D, right upper panel). In MCF-7 cells transduced with Ad-GREB1, the metabolic activity as measured by AlamarBlue was also increased by 1.5 fold compared to Ad-CMV-null transfected controls (Figure 4D, right lower panel), suggesting that GREB1 may function as a growth promoter in breast cancer and promote cell proliferation. It is noteworthy that the transfection efficiency varied among different breast cancer cell lines. For example, the transfection efficiency in E2-deprived MCF-7 cells (21- fold in Figure 4D, middle upper panel) is slightly lower than in ER-negative cells such as MDA-MB-231 (63-fold in Figure 4A, right upper panel), MDA-MB-453 (45-fold in Figure 4B, right upper panel) and MDA-MB-468 (40-fold in Figure 4C, right upper panel).

**Figure 4:** Overexpression of GREB1 promotes cell proliferation and increases the clonogenic ability of breast cancer cells. MDA-MB-231, MDA-MB-453, MDA-MB-468 and estrogen depleted MCF-7 for 3 days were infected with Ad-CMV-null and Ad-GREB1 at an MOI of 10 respectively. The cells transduced with Ad-GREB1 expressed high GREB1 mRNA levels, whereas GREB1 was at extremely low detectable level in all cells including estrogen deprived MCF-7 asynchronous cultures (Figure 4D, middle upper panel), MDA-MB-231 (Figure 4A, right upper panel), MDA-MB-453 (Figure 4B, right upper panel), and MDA-MB-468 (Figure 4C, right upper panel) cell cultures transduced with empty vector. The soft agar assay was used as a measure of anchorage independent growth. The ability of MDA-MB-231 (Figure 4A, left panel), MDA-MB-453 (Figure 4B, left panel), MDA-MB-468 (Figure 4C, left panel), and MCF-7 (Figure 4D, middle lower panel) to grow in soft agar is substantially enhanced 1.9-, 2.2-, 1.7- and 2.0- fold following GREB1 transfection. We next tested E2 deprived MCF-7 cells for the effects of GREB1 on cell proliferation. The growth rate in MCF-7 cells treated with E2 is 3.5 fold higher than in estrogen depleted, quiescent controls. Transfection with the SiGREB1 had significant effect on cells treated with E2, as showed here that cell proliferation was completely abolished (Figure 4D, right upper panel). In MCF-7 cells transduced with Ad-GREB1, the metabolic activity as measured by AlamarBlue was also increased by 1.5 fold compared to Ad-CMV-null transfected controls (Figure 4D, right lower panel). The transfection efficiency in E2-deprived MCF-7 cells (21- fold in Figure 4D, middle upper panel) is a little lower than those of ER-negative cells such as MDA-MB-231 (63-fold in Figure 4A, right upper panel), MDA-MB-453 (45-fold in Figure 4B, right upper panel) and MDA-MB-468 (40-fold in Figure 4C, right upper panel). Figure 4E showed the little higher basic expression level of GREB1 in E2-deprived MCF-7 cells than other cells. Data are shown as mean ± SD. *P<0.05; **P<0.01.

### IL6/STAT3 Modulates Estrogen-induced GREB1 Transcriptional Activity in Breast Cancer Cells

Previous reports indicated that STAT3 acts downstream of HER2 [23], [24]. STAT3 is tyrosine phosphorylated through the interleukin-6 (IL-6)/glycoprotein 130/Janus kinase pathway in breast cancer [25]. Interestingly, we found several STAT3 binding sites TT(N4)AA and TT(N5)AA located in the human GREB1 promoter region (http://www.cbrc.jp/research/db/TFSEARCH.html), which incidentally also contains three consensus EREs. STATs and ER can physically interact in vivo [26]. Based on this information, we hypothesize that STAT3 may physically connect with ER to repress GREB1 transcriptional activity or compete with ER for DNA binding sites within the multiple estrogen inducible enhancer regions of GREB1, resulting in decreased or non-detectable GREB1 expression. To test this hypothesis, we first assayed the effects of IL-6 on estrogen-induced GREB1 gene expression. Total RNA was extracted from estrogen-deprived MCF-7 cells for 3 days followed by exposure to E2 for 48 h. A region specific to GREB1a transcripts was amplified by real-time polymerase chain reaction (qPCR). The results show that E2 treatment increases GREB1 mRNA levels by approximately 43-fold after 48 h treatment (Figure 5A). ICI abolishes E2-induced GREB1 expression. As expected, IL-6 has an inhibitory effect on GREB1 expression, which inhibits GREB1 expression by approximately 44% (Figure 5A). IL-6 is known to activate many downstream signaling pathways, we thus asked whether the inhibitory effect of IL-6 on E2-induced GREB1 transcription is due to JAK/STAT3 cascade activation. Therefore, we designed the experiments to test what would happen to E2-mediated GREB1 induction if STAT3 gene was knocked down or kept constitutively active. Transfection with STAT3 siRNA (SiSTAT3) duplexes increased E2 induced expression of GREB1 (Figure 5B) whereas transfection with constitutively active STAT3 vector (STAT3-C) suppressed E2 induced expression of GREB1 (Figure 5C). We then asked how IL-6 affects transcriptional activation of GREB1. The construct was established by cloning a 1.7-kb fragment containing ERE1 and the GREB1a promoter region into pGL3 reporter plasmid, followed by inserting ERE2 and ERE3 upstream of ERE1. The DNA fragment contains all three EREs. MCF-7 cells were estrogen deprived for 3 days before transfection with 0.5 µg luciferase GREB1 promoter-reporter construct and 0.1 µg phRL-SV40 Renilla internal control (Promega). The following day, transfected cells were continued to befed with medium containing 1 nM E2 and 10 ng/ml IL-6 for a further 24 h before lysis and measurement of luciferase activity using the Dual Luciferase Assay kit (Promega). As shown in Figure 5D, E2 treatment increases luciferase activity by approximately 37-fold over the control. Estrogen receptor antagonist ICI 182,780 blocks the E2-mediated GREB1 induction, confirming that the increased GREB1 is due specifically to the E2 stimulation. Interestingly IL-6 inhibits E2-induced GREB1 transcriptional activity by approximately 38%. To determine the most efficient concentration for IL-6, hormone-starved MCF-7 cells were treated with various concentrations of IL-6 (0∼100 ng/ml) for 24 h. As shown in Figure 5E, inhibition of of E2-mediated GREB1 activity by IL-6 peaked at 10 ng/ml. In the subsequent time course experiments, cells were treated with 10 ng/ml IL-6 for 0, 10, 20, 30 min until 24 h, and the resulting inhibition of E2-induced GREB1 level was similarly analyzed. We observed that the effects on the reduction of GREB1 by IL-6 did not vary significantly from 1 h to 24 h, GREB1 transcriptional activity indicated by GREB1 luciferase activity was significantly diminished at each time point compared to E2 stimulation alone (*P<0.05, compared to E2 stimulation alone). Interestingly, pretreatment with IL-6 for less than half an hour significantly dampered the antagonistic function of IL-6 on suppression of E2-induced GREB1 (Figure 5F). To determine if the expression levels of STAT3 would have any effect on the transcriptional activity of GREB1, MCF-7 cells were cotransfected with a GREB1 luciferase reporter construct, a STAT3 constitutively expressing vector (STAT3-C), and a control vector, respectively. Some samples were treated with E2 as indicated before assaying for luciferase activity. As shown in Figure 5G, STAT3-C decreases GREB1 transcription by approximately 39%.

**Figure 5:** IL6/STAT3 modulates estrogen-induced GREB1 transcriptional activity in breast cancer cells. E2 treatment increases GREB1 mRNA levels by approximately 43-fold after 48 h treatment (Figure 5A). ICI abolishes E2-induced GREB1 expression. IL-6 has an inhibitory effect on GREB1 expression, which inhibits GREB1 expression by approximately 44% (Figure 5A). Transfection with STAT3 siRNA (SiSTAT3) duplexes increased E2 induced expression of GREB1 (Figure 5B) whereas transfection with constitutively active STAT3 vector (STAT3-C) suppressed E2 induced expression of GREB1 (Figure 5C). Figure 5D to 5G, MCF-7 cells were estrogen deprived for 3 days before transfection with 0.5 µg luciferase GREB1 promoter-reporter construct and 0.1 ug phRL-SV40 Renilla internal control. The following day, transfected cells were refed with medium containing 1 nM E2 and 10 ng/ml IL-6 for a further 24 h before lysis and measurement of luciferase activity. As shown in Figure 5D, E2 treatment increases luciferase activity by approximately 37-fold over the control. Estrogen receptor antagonist ICI blocks the E2-mediated GREB1 induction. IL-6 inhibits E2-induced GREB1 transcriptional activity by approximately 38%. To determine the best efficient concentration for IL-6, hormone-starved MCF-7 cells were treated with various concentrations of IL-6 (0∼100 ng/ml) for 24 h. Figure 5E shows that the maximum reduction of E2-mediated GREB1 activity is seen at 10 ng/ml, the inhibitory effects are decreased regardless of whether the doses are further increased or decreased throughout the experiment. In time course experiments, cells were treated with 10 ng/ml IL-6 at indicated time,. Pretreatment with IL-6 for less than half an hour dampered the antagonist function of IL-6 on suppression of E2-induced GREB1 greatly (Figure 5F). MCF-7 cells were then cotransfected with a GREB1 luciferase reporter construct, a STAT3 constitutively expressing vector (STAT3-C) and control vector respectively. The samples were treated with E2 as indicated before assaying for luciferase activity. As shown in Figure 5G, STAT3-C decreases GREB1 transcription by approximately 39%. Data are shown as mean ± SD. *P<0.05; **P<0.01.

### STAT3 physically Interacts with ERα

To confirm whether there is a physical interaction between STAT3 and ERα, we transfected 293T cells with FLAG-tagged STAT3-C alone or together with ERα. 48 h after transfection, cells were treated with 1 nM E2 for 3 h. Cell lysates were then immunoprecipitated with anti-ERα and immunoblotted with anti-FLAG (Figure 6A). Immuno-complex was probed with anti- ERα antibody as internal loading control. Norml rabbit IgG served as negative control. Cell lysates were also immunoprecipitated with anti-FLAG from two different commercially available sources (Millipore and Sigma respectively), followed by immunoblotted with anti-ERα as indicated in Figure 6B. Immuno-complex was probed with anti- FLAG antibody as internal loading control. The results from Figure 6 indicate that STAT3 indeed directly interacts with ERα.

**Figure 6:** STAT3 physically interacts with ERα. To confirm whether there is a physical interaction between STAT3 and ERα, we transfected 293T cells with FLAG-tagged STAT3-C (2 µg) alone or together with ERα (2 µg). 48 h after transfection, cells were treated with 1 nM E2 for 3 h. Cell lysates were immunoprecipited with anti-ERα and immunoblotted with anti-FLAG as shown in Figure 6A. Figure 6B showed that cell lysates were first immunoprecipitated with anti-FLAG from two different commercially available resources (Millipore and Sigma) respectively followed by immunoblotted with anti-ERα. The results from Figure 6 indicate that STAT3 indeed directly interacts with ERα.

## Discussion

Whether tamoxifen acts as an agonist or antagonist is intimately related to AF domain activation. AF-1 activity is regulated by phosphorylation and is ligand-independent; AF-2 is the ligand-binding domain (LBD). AF-1 and AF-2 act synergistically under most conditions, but each can also act independently. When tamoxifen binds to the ERα LBD, the changes in structural conformation prevent binding of co-activators, suppressing AF-2 promoted transcription. In this situation, tamoxifen acts as an antagonist. In genes where AF-2 function is redundant and transcription is driven by the AF-1 region, tamoxifen may act as an agonist. Multiple mechanisms have been proposed as responsible for tamoxifen resistance in breast cancer [6]. Among them, the alterations in ERα expression/function contribute greatly to resistance to tamoxifen. ER/PgR negative tumors do not respond to tamoxifen. In ER positive breast cancer patients, the levels of ERα expression reflect the possibility of benefit from endocrine therapy [54]. Transcriptional silencing of ERα by DNA methylation has been well documented in patients with recurrent breast cancer who have received tamoxifen therapy, whereas mutations within the open reading frame of ER in patients are not common although some mutations in the ER have been examined in resistant cell lines [6], [54]. The majority of ER-positive patients still expresses quite high levels of ERα at the time disease progresses and develops acquired tamoxifen resistance [17], [54]. Phosphorylation of ERα (Ser118) and sequential activation of its downstream pathway induced by tamoxifen has been reported to contribute to the development of endocrine therapy resistance and predict poor prognosis [54].

While ER expression status has important treatment and prognosis implication in breast cancer patients, ER alone is not perfectly correlated with hormonal response [55]. To determine the possibility of GREB1 functions as a surrogate marker for ER in clinical situation, we analyzed the GREB1 expression status in normal breast tissues, ER-positive and ER-negative breast cancer tissues using Oncomine public database and gene microarray data analysis tool [32], [33]. Our results show that GREB1 mRNA is highly expressed in breast carcinomas than normal breast tissues (T-test: 4.815; P-value: 2.1E-5), GREB1 mRNA is significantly overexpressed in ER-positive breast cancer patients compared to that of ER-negative patients (Figure 2) [34], [35], [36], [37], [38], [39], [40], [41], [42], [43], [44], [45], [46], [47]. Furthermore, analysis of GREB1 mRNA in 225 patients from the Tamoxifen (TAM) arm of 89-30-52 indicates that GREB1 can serve as an independent predictor of good disease-free survival in Tamoxifen-treated patients in ways even more reliable than ER or PgR, which itself has historical precedence as a clinical prognosticator in breast cancer patients in response to endocrine therapy (Table 1) [8], [51], [52]. This conclusion is further supported by a patient survival analysis to correlate GREB1 gene expression and relapse free survival for 2898 breast cancer patients (www.kmplot.com) where loss or reduced level of GREB1 is strongly predictive of worse disease outcome for all breast cancer patients in general, and for ER+, and ER+ endocrine treated patients in particular (Figure 2C to 2E). Based on these data, we believe that GREB1 protein may have a great potential to be a new biomarker not only for predicting ER and/or PgR status, but also for predicting Tomoxifen treatment response in breast cancer patients.

The role of GREB1 in regulating hormone-related cancer including mammary carcinoma proliferation has been investigated for some time [28], [56]. However, no studies have systemically explored the role of GREB1 in cellular proliferation and cell growth [28], [56]. In the results presented here, we showed for the first time that increased levels of GREB1 have the growth advantage seen in breast tumors, with a 150% increase in MCF-7 cells expressing Ad-GREB1 than cells containing control vector at time points of 48 h after infection (Figure 4D, right lower panel). We also showed that RNAi directed against GREB1 significantly decreased the growth rate of MCF-7 cells (Figure 4D, right upper panel). We then tested whether adeno-GREB1-mediated increase in GREB1 expression could influence the ability of different breast cancer cell lines including MCF-7, MDA-MB-231, MDA-MB-453, and MDA-MB-468 to form colonies in soft agar. Adeno-directed increase in GREB1 resulted in a significant increase (about 170%–220%) in colony formation in all four breast cancer cell lines regardless of ER status (Figure. 4). These results clearly demonstrate that increased GREB1 levels enhance the clonogenic ability of breast cancer cells. In another word, elevation of GREB1 levels has substantial effects on the transformed phenotype of breast cancer cells. The tumorigenesis assays in which GREB1-expressing cells exhibit a greater capability to display a transformed phenotype are important since GREB1-mediated signaling pathways may be useful in inhibiting tumor formation in vivo. A slightly higher basic expression level of GREB1 in E2-deprived MCF-7 cells as shown in Figure 4E may cause difficulty in introducing exogenous GREB1 gene into these cells and may account for the higher transfection efficiency in MDA-MB-231, MDA-MB-453 and MDA-MB-468 cells than E2-deprived MCF-7 cells.

IL-6 is a multifunctional cytokine that has important roles in the immune system, hematopoiesis, and acute phase reactions [27]. In addition, IL-6 has been found to inhibit the growth of human breast cancer cells in vitro in the presence of E2 and modulate the ER and PgR [57]. In the present study, the breast cancer growth promoter, E2-induced GREB1 transcriptional activity was found to be significantly diminished by IL-6 compared to E2 stimulation alone (Figure 5F). Clinical studies showed that patients with STAT3 nuclear expression had a significantly improved 5-year survival, patients with phospho-STAT3 (Tyr705) nuclear expression had a significantly improved survival at both short-term (5-year ) and long-term (20-year) survival [58], and phosphor-STAT3 (Tyr705) is a marker for improved overall survival independent of other prognostic markers [58]. The glycoprotein 130 (gp130) receptor and gp130-associated JAKs are known mediators of STAT3 phosphorylation [25]. JAK2 was recently found to negatively regulate expression of endogenous ERα target genes, such as GREB1 and pS2 [59]. JAK2 mediated downregulation of ERα via the ubiquitin-proteasome pathway. This negative feedback modulation of ERα is physiologically essential to limit estrogen action in target tissues [59]. It is therefore not surprising for us to show here that IL-6 as well as its downstream pathway molecules STAT3 inhibit the transcriptional expression of E2-target gene GREB1. It is noteworthy in our observation that GREB1-expressing MDA-MB-231 and MDA-MB-468 cells still displayed enhanced ability to form colonies in soft agar even though these cells constitutively expressed tyrosine-phosphorylated STAT3 [25]. This indicates that endogenous phosphor-STAT3 is unable to completely offset the exogenous GREB1 function in these two cell lines. ER has been found to interact with some STAT proteins [26], [27]. Early research on the cross-talk between ER and STAT5a indicated that cross-talk between ER and STAT5a was through a direct physical association between the two proteins, and their C-termini were mainly responsible for this interaction [26]. We provided evidence here that the inhibitory function of STAT3 on GREB1 expression was also caused by a direct physical interaction between STAT3 and ER, and subsequently in the presence of E2, the low receptor level of ER leads to reduced transcriptional activity of ER-target genes such as GREB1.

GREB1 is a primary E2 target gene and is strongly and sustainably induced by estrogen [28], [29], [30], [31]. We show that GREB1 expression is associated with ERα expression in breast cancer cell lines and breast cancer tissues. ERα directly controls GREB1 expression, and GREB1 is required for breast cancer cell growth. Clinically, like ER status, the loss or reduced expression of GREB1 is predictive of worse therapeutic outcome and decreased relapse free survival. Overall, our studies provide new insight into the biological function of GREB1 and its role in the pathogenesis of breast cancer.

## Materials and Methods

### Antibodies and Reagents

Monoclonal antibody against GREB1 was obtained from ProMab Biotechnologies Inc (Richmond, CA). Antibody to β-actin was obtained from Sigma-Aldrich. All secondary antibodies used for Western blot were purchased from Calbiochem. GREB1 siRNA, STAT3 siRNA and control siRNA were purchased from Dharmacon (Lafayette, CO). The GREB1 promoter-luciferase construct was obtained as a generous gift from Joyce Slingerland (Department of Medicine, University of Miami, Miami, FL). Constitutive active STAT3 construct (STAT3-C) is kindly provided by Jacqueline F. Bromber (Department of Medicine, Memorial Sloan-Kettering Cancer Center, New York, NY).

### Microarray Analysis from Meta-analysis of Oncomine Database

The expression of GREB1 transcript in breast normal and cancer tissues was obtained from meta-analysis of cancer gene microarray meta-analysis public database [32], [33]. Statistical analysis of differences was performed using Oncomine algorithms to account for the multiple comparisons among different studies similar to a meta-analysis as previously described [60].

### Brest Cancer Cell Lines and Culture Conditions

Breast carcinoma cell lines MCF-7, MDA-MB-231, MDA-MB-453 and MDA-MB-468 were from American Type Culture Collection (ATCC) and were maintained and growth assays were performed as described previously [28], [61]. For defined estrogen culture experiments, cells were washed and grown in steroid depleted media (phenol red-free IMEM supplemented with 5% charcoal stripped calf bovine serum-Valley Biomedical Products, VA).

### SiRNA Transfection

Small interfering RNA (siRNA) duplexes (total four pairs) of GREB1 and STAT3 were designed and purchased from Dharmacon (Lafayette, CO). A scrambled siRNA, with no homology to any known sequence was used as control. Hormone-depleted MCF-7 cells were transfected with 100 nM specific siRNA or control using Lipofectamine™ reagent (Invitrogen, Carlsbad, CA) in serum free OptiMEM-1 medium (Invitrogen) according to the manufacture’s instruction. After six hours of transfection, MCF-7 cells were split into two groups and grown in 10% CCS for another 24 h, then the cells were treated with 1 nM E2 or 0.01% ethanol; MDA-MB-231, MDA-MB-453, and MDA-MB-468 cells were grown in 10% FBS for 24 h. All studies were done in triplicates.

### Real-time RT-PCR Analysis

Cell pellets were stored in Trizol reagent and homogenized in fresh Trizol. Total RNA were isolated from cells using an RNeasy Mini Kit (Qiagen, Valencia, CA). cDNA were synthesized from the isolated RNA using iScript cDNA Synthesis Kit (Bio-Rad Laboratories, Inc). Reverse transcription was performed by using random hexamers at 25°C for 5 minutes, 42°C for 30 minutes, and 85°C for 5 minutes. Quantitative PCR were performed using iQ SYBR Green Supermix (Bio-Rad Laboratories, Inc.) in a CFX96 Real-Time PCR System machine (Bio-Rad Laboratories, Inc). The data was analyzed using CFX96 Real-Time PCR System (Bio-Rad Laboratories, Inc). Primer sequences for the human GREB1 are: GREB1a-F: 5′-AAATCGAGGATGTGGAGTG-3′, GREB1a-R: 5′-TCTCACCAAGCAGGAGGA-3′.

### Luciferase Reporter Gene Assay

MCF-7 cells were transfected using lipofectamine 2000 (Invitrogen) with 0.75 µg of GREB1 promoter-luciferase construct together with 100 µg of pRL-TK, a cytomegalovirus-Renilla vector to control transfection efficiency. The amount of total DNA transfected was equalized with the appropriate amounts of control vectors. After transfection at different indicated points, cells were harvested and lysed in reporter lysis buffer (Promega, Madison, WI). Luciferase activity was determined by using the Dual Luciferase Kit (Promega) and a luminometer (Turner Design, Sunnyvale, CA) according to the manufacturer’s recommendation. All luciferase results were normalized to Renilla activity from the co-transfected pRL-TK plasmid. The data for luciferase activity was expressed as fold induction with respect to control cells and was the mean ± standard error of triplicate samples.

### Immunoprecipitation and Western Blot

Cells were lysed with lysis buffer (50 mmHEPES, 150 mmNaCl, 1.5 mm MgCl2, 1 mm EGTA, 10% glycerol, 1% Nonidet P-40, 100 mm NaF, 10 mm sodium pyrophosphate, 0.2 mm sodium orthovanadate, 1 mm phenylmethylsulfonyl fluoride, 10 µg/ml aproptinin, and 10 µg/ml leupeptin). After centrifugation, protein lysates (50 µg) or the immunoprecipitates from cell lysates (500 µg) were separated on a 4–15% gradient gel (Bio-Rad Laboratories) and transferred to a nitrocellulose membrane and immunoblotted with the appropriate antibodies. The membrane was blocked in 5% nonfat dry milk in TBST for 1 h at room temperature and incubated with mouse antibody to human GREB1 (ProMab Biotechnologies Inc) at a dilution of 1∶1000 in TBST +2.5% nonfat dry milk, followed by horseradish peroxidase-conjugated antimouse secondary antibody (Amersham) at a dilution of 1∶2,000. Immunoblots were reprobed with β-actin monoclonal antibody to confirm equal loading. The expression levels of GREB1 and β-actin detected by immunoblotting were quantitated using the ImageQuant program (Bio-Rad) for the integrated density of each band. Western blot assays were conducted in duplicate for each sample and the mean value was used for the calculation of protein expression levels.

### AlamarBlue Assay

After trypsinization, the indicated cancer cell lines were counted and resuspended to a final concentration of 1×10^4^ cells/ml. A 100 µl aliquot of the cell suspension were seeded per well in 96 well plates. The stock solution of AlamarBlue was aliquoted and stored and protected from light at −20°C. 20 µl of AlamarBlue was added to each well at 48 h and the 96 well plates were returned to the incubator for 6 h. Absorbance was monitored with excitation at 570 nm and emission at 600 nm using a CytoFluorTM 2300 plate reader and the software CytoFluorTM 2300 v. 3A1 (Millipore Co, Bedford, MA, USA).

### Anchorage-Independent Growth Assays

MCF-7 cells were hormone starved for 3 days in PRF IMEM containing 10% CS-FCS (HyClone). MDA-MB-231, MDA-MB-453 and MDA-MB-468 cells were grown in regular media containing 10% FBS. At 2 days after transfection, cells (300 cells per well) transfected with indicated plasmids were mixed with tissue culture medium containing 0.7% agar to result in a final agar concentration of 0.35%. Then 1 ml samples of this cell suspension were immediately plated in six-well plates coated with 0.6% agar in tissue culture medium (2 ml per well) and cultured at 37°C with 5% CO2. After 2 weeks, tumor cell colonies measuring at least 150 µm were counted from three replicates per treatment under a dissecting microscope.

### Immunoflurescence Microscopy

Cells grown in monolayer cultures were fixed with 4% paraformaldehyde in phosphate-buffered saline (PBS), permeabilized with 0.2% Triton X-100, and blocked with 10% fetal calf serum prior to antibody staining. Staining by anti-GREB1 antibody (1∶100) was visualized with corresponding Alexa Fluor® 555-labeled secondary antibody. Cover slips were mounted onto slides with Vectashield mounting medium with DAPI (H-1200; Vector Laboratories Inc). Fluorescent images were collected by using a Zeiss LSM510 confocal microscope, and images were captured with LSM software, version 2.3.

### Immunohistochemistry Staining

Breast tumor tissue microarrays (TMA) were provided by Tissue Array Networks (http://Tissue-Array.Net). Slides containing formalin-fixed, paraffin-embedded samples were deparaffinized, hydrated in water, and subjected to antigen retrieval in 10 mM citrate buffer, pH 6.0. Immunostaining was performed as described previously with some modifications [62]. Briefly, slides were probed with GREB1 antibody at a dilution of 1∶100 for 1 hour, then probed with secondary antibody for another one hour. The reaction products were finally visualized by immersing slides in 3, 3-diaminobenzidine tablet sets (Sigma Fast, Sigma) and counterstained with hematoxylin. The anti-ER antibody (clone 1D5, dilution 1∶100; Dako) used is FDA approved [63]. TMAs were reviewed and scored by two pathologists (C.R. G. and M.J.).

### Patient Survival Analysis

An online database [Gyorffy et al 2010] was used to assess relevance of GREB1 expression to relapse free survival. The database was established using gene expression data and survival information of 1,809 patients (recently increased to 2898 patients) downloaded from Gene Expression Omnibus (GEO) (Affymetrix HGU133A and HGU133+2 microarrays). Briefly, GREB1 gene was entered into the database (http://kmplot.com/breast/) to obtain Kaplan-Meier survival plots where the number-at-risk is indicated below the main plot. Hazard ratio (and 95% confidence intervals) and logrank P were calculated and displayed on the webpage.

### Statistical Analysis

Results were expressed as mean ± SEM of at least 2 independent experiments done in triplicate. Paired t-test or ANOVA tests were performed for data analysis, and significant difference was defined as p<0.05.
